This article has been retracted.

# Stereochemical Insignificance Discovered in *Acinetobacter baumannii* Quorum Sensing

**DOI:** 10.1371/journal.pone.0037102

**Published:** 2012-05-22

**Authors:** Amanda L. Garner, Sook Kyung Kim, Jie Zhu, Anjali Kumari Struss, Richard Watkins, Brent D. Feske, Gunnar F. Kaufmann, Kim D. Janda

**Affiliations:** 1 Departments of Chemistry and Immunology and Microbial Science, The Scripps Research Institute, La Jolla, California, United States of America; 2 The Skaggs Institute for Chemical Biology, The Scripps Research Institute, La Jolla, California, United States of America; 3 The Worm Institute for Research and Medicine, The Scripps Research Institute, La Jolla, California, United States of America; 4 Department of Chemistry, Armstrong Atlantic State University, Savannah, Georgia, United States of America; University of Wisconsin, Food Research Institute, United States of America

## Abstract

Stereochemistry is a key aspect of molecular recognition for biological systems. As such, receptors and enzymes are often highly stereospecific, only recognizing one stereoisomer of a ligand. Recently, the quorum sensing signaling molecules used by the nosocomial opportunistic pathogen, *Acinetobacter baumannii*, were identified, and the primary signaling molecule isolated from this species was *N*-(3-hydroxydodecanoyl)-l-homoserine lactone. A plethora of bacterial species have been demonstrated to utilize 3-hydroxy-acylhomoserine lactone autoinducers, and in virtually all cases, the (*R*)-stereoisomer was identified as the natural ligand and exhibited greater autoinducer activity than the corresponding (*S*)-stereoisomer. Using chemical synthesis and biochemical assays, we have uncovered a case of stereochemical insignificance in *A. baumannii* and provide a unique example where stereochemistry appears nonessential for acylhomoserine lactone-mediated quorum sensing signaling. Based on previously reported phylogenetic studies, we suggest that *A. baumannii* has evolutionarily adopted this unique, yet promiscuous quorum sensing system to ensure its survival, particularly in the presence of other proteobacteria.

## Introduction

Bacteria exploit many mechanisms to gain advantage over environmental competitors and confer protection on themselves to ensure their survival. In Gram-negative bacteria, a class of autoinducers, the *N*-acyl-homoserine lactones (AHLs), have been identified as key mediators for cell-to-cell signaling, or quorum sensing, necessary for virulence factor expression and biofilm formation [1]–[3]. For example, in *Pseudomonas aeruginosa*, quorum sensing is mediated by two AHLs, *N*-(3-oxododecanoyl)-L-homoserine lactone **1** (3-oxo-C_12_-HSL) and *N*-butyryl-L-homoserine lactone **2** (Figure 1A) [4]–[6]. Similar to *P. aeruginosa*, *Acinetobacter baumannii* is also a nosocomial opportunistic pathogen and accounts for ∼10% of hospital-acquired infections [7]–[9]. This species has been linked to numerous types of clinical manifestations including wound, bloodstream and urinary tract infections, ventilator-acquired pneumonia, septicemia and necrotizing fasciitis [7]–[9]. Importantly, *A. baumannii* has been found to be prevalent in a large number of infection cases in wounded military personnel returning from combat in Iraq and Afghanistan earning it the nickname “Iraqibacter" [8], [9]. *A. baumannii* has proved to be a particularly daunting challenge as the bacteria easily adapt to variable conditions and are able to survive even in dry, desiccated environments [9]. Moreover, many strains of this species are gaining multidrug resistant phenotypes, including resistance to β-lactam antibiotics, quinolones and colistin; thus, new therapies are needed to target such infections [7], [9].

**Figure 1:** *N*-Acyl-homoserine lactone autoinducers. A, *P. aeruginosa* autoinducers. B, *A. baumannii* autoinducer.

Recently, an autoinducer synthase (AbaI) and corresponding AHL signaling molecules were reported for *A. baumannii* [10]. The primary AHL isolated from this species was identified as *N*-(3-hydroxydodecanoyl)-L-homoserine lactone (**3**, 3-OH-C_12_-HSL, Figure 1B) by mass spectrometry and confirmed with a synthetic sample [10]. Although little is known regarding factors required for biofilm formation and virulence factor expression in *A. baumannii* [11], this process was found to be impaired in an *abaI*::Km mutant incapable of producing AHLs [10] indicating that quorum sensing signaling molecules, including AHL **3**, may play a role in this process.

To date, 3-hydroxy-substituted AHLs have been identified in a limited number of bacterial species [12]–[16]. With respect to AHL **3**, this autoinducer has previously been identified as a quorum sensing signaling molecule in *Vibrio scophthalmi* [17], *Yersinia pseudotuberculosis* [18] and *Acidithiobacillus ferrooxidans* [19], each of which is unrelated to *A. baumannii*. Interestingly, despite the presence of a stereocenter at the 3-hydroxy position in **3**, chirality requirements at this site in AHL **3** produced by *A. baumannii* have remained cryptic; however, the stereochemistry of the 3-OH position has been defined in 3-OH AHLs from other species [15], [16], [20], [21]. In most of these prior cases, the (*R*)-stereoisomer was identified as the natural stereoisomer and was found to exhibit greater autoinducer activity than the corresponding (*S*)-stereoisomer [15], [16], [20], [21]. The detection of (*R*)-stereochemistry at this position is not surprising, as AHL biosynthesis is believed to be stereoselective with respect to the 3-OH stereocenter, and FabG, the β-ketoacyl acyl carrier protein reductase of the fatty acid biosynthetic pathway, has been shown to selectively produce (*R*)-hydroxy substituents following reduction of the corresponding β-ketoacyl moieties [22]–[24]. Moreover, lactone stereochemistry has already been shown to be critical for autoinducer activity [25]. Thus, since molecular recognition in biological systems is generally highly stereospecific, we were interested in deciphering the stereochemical requirements at this position. To complement the lactone-focused stereochemical explorations, herein, we describe our efforts to synthesize each diastereomer of AHL **3** and examine their impact on quorum sensing in *A. baumannii*. From our studies, we have uncovered a case where stereochemical integrity does not affect the biological signaling process, thus, providing an example where a stereochemical center appears non-critical for biological activity.

## Results

### Synthesis of AHL 3 Autoinducers

Our studies commenced with the chemical syntheses of both diastereomers of AHL 3 (Figure 2) (see Supporting Information for experimental detail). The syntheses began with commercially available fatty acid 4, which was first activated with DCC followed by nucleophilic displacement of the resultant activated ester with Meldrum's acid and coupling with l-homoserine lactone 5 to yield AHL 1. Enantioselective reduction of the 3-oxo-position was performed using Corey-Bakshi-Shibata reduction conditions to obtain AHL diastereomers 3a and 3b [26]. Mosher ester analysis [27] was used to confirm the stereochemical integrities of AHLs 3a and 3b (see Supporting Information for experimental detail and assignment: Scheme S1, Table S1, Figures S1, S2, S3, S4, S5, and S6). Since it was previously demonstrated that the stereochemistry of the lactone ring is key for activity in *P. aeruginosa* [28] among other Gram-negative bacteria [29], only the l-homoserine lactone ring was examined at this position.

**Figure 2:** Synthesis of (*R*)-3-OH-C_12_-l-HSL (3a) and (*S*)-3-OH-C_12_-l-HSL (3b).

### Characterization of AHL 3 Autoinducers in *A. baumannii*

With the diastereomerically pure lactones in hand, we examined their impact as autoinducers in *A. baumannii*. Autoinducer assays were conducted using an *abaI*::*lacZ* mutant *A. baumannii* strain wherein the *abaI* promoter is fused with a *lacZ* gene [10]. In this assay, since the *abaI* gene is activated in a positive feedback loop by an AbaI-dependent AHL signal, successful autoinducers will promote expression of lacZ. Mutant *A. baumannii* were treated with varying concentrations of AHLs **3a** and **3b** (0–100 µM), and β-galactosidase activity was measured using a luminescence-based assay (see Supporting Information). Unexpectedly, as Figure 3A shows, AHL diastereomers **3a** and **3b** exhibited nearly the same autoinducer activity with EC_50_ values of 0.67 ± 0.06 µM and 0.82 ± 0.06 µM, respectively, and no statistical significance was found between these values (p  =  0.3471). Of further significance, the activities of **3a** and **3b** were also nearly identical at lower, more physiologically relevant concentrations (Figure 3C). This is important, as receptors have typically evolved to specifically recognize one stereochemical form of a molecule. To underscore the relevance of this finding, in *Vibrio harveyi* [16] and *Rhizobium leguminosarum* [20], [21], their corresponding 3-OH AHLs were identified as possessing (*R*)-3-OH stereocenters, and in each case, the unnatural (*S*)-isomer exhibited little to no autoinducing activity. Moreover, previous studies in the AHL biosensor strains *E. coli* MT102 (pJBA132) and *Pseudomonas putida* F117 (pKR-C12) showed a difference in potency between (*R*)-3-OH-C_8_-HSL and (*S*)-3-OH-C_8_-HSL, albeit only at concentrations beyond 10 µM [15]. A similar finding was also reported earlier in *Erwinia carotovora*, and a>3-fold difference in activity was noted between the two diastereomers of 3-OH-C_6_-HSL [29]. Thus, our findings in *A. baumannii* appear to be unique.

**Figure 3:** Autoinducer activities of AHL derivatives in an *abaI*::*lacZ* mutant *A. baumannii* strain. Values shown are relative luminescence units normalized with respect to cell viability (OD_600_). A, Autoinducer activities from 0–100 µM. Closed circle  =  **3a**. Open circle  =  **3b**. Closed triangle  =  **1**. Square  =  **6**. Open triangle  =  3-oxo-C_12_-d-HSL. B, Structure of *N*-(3-dodecenoyl)-l-homoserine lactone (**6**). C, Enhanced view of autoinducer activity of **3a** and **3b** at lower concentrations. Closed circle  =  **3a**. Open circle  =  **3b**. EC_50_ and p values determined using GraphPad Prism v5.0b for Mac OS X.

In addition to AHLs **3a** and **3b**, although not produced by AbaI, AHL **1** was also found to exhibit autoinducer activity, but to a lesser extent (Figure 3A). Stereochemistry of the lactone ring, as expected, was found to be vital, and 3-oxo-C_12_-d-HSL showed diminished autoinducer activity (Figure 3A) in comparison to AHL **1**. We also examined the effect of treatment with *N*-(3-dodecenoyl)-l-homoserine lactone (**6**, Figure 3B), a possible elimination product common to both AHLs **3a** and **3b**; however, no activity was observed with this compound (Figure 3A). In sum, these results indicate that an oxygen heteroatom is required at the 3-position, possibly due to hydrogen bonding interactions within the AHL **3** binding site in AbaR, and lactone stereochemistry is critical as previously found in other bacterial species utilizing AHLs.

To determine whether AHLs **3a** and **3b** are acting on the same or different receptors in *A. baumannii*, the mutant strain was treated with varying concentrations of a 1∶1 mixture of AHLs **3a** and **3b**. As Figure 4 shows, no change in autoinducer activity was observed with this epimeric mixture. These results indicate that AHLs **3a** and **3b** act on the same receptor in an equipotent manner. This finding adds to the curiosity of our study, and may demonstrate that the lactone configuration (i.e., the “head") is more crucial for receptor binding and that “tail" substitution may provide only minor interactions within the AbaR AHL binding site, as both 3-hydroxy configurations and the 3-oxo moiety showed activity.

**Figure 4:** Autoinducer activity of a 1∶1 mixture of 3a and 3b. Values shown are relative luminescence units normalized with respect to cell viability (OD_600_). Square  =  1∶1 **3a∶3b**. Closed circle  =  **3a**. Open circle  =  **3b**.

### Stability Studies of AHL 3 Autoinducers

To ensure that the added AHL compounds were not being chemically modified during the course of our assay, the stability and chemical integrity of AHL **3** was assessed. It has been well documented that AHLs undergo lactone hydrolysis over extended incubation periods under physiological conditions [30]. Additionally, our group uncovered an additional side reaction of AHL **1**, namely the formation of a tetramic acid via an intramolecular Claisen-like condensation reaction [31]. To determine the stability and possible side products of AHL **3**, a derivative of this compound containing an aromatic moiety at the tail end (see Supporting Information and Scheme S2 for experimental detail) was used to aid in HPLC and LC-MS analyses. The compound was assayed in phosphate buffered saline (PBS) (pH 7.4) at 37°C over a period of 36 h. From this study, the half-life of AHL **3** was found to be approximately 20 h, which is similar to that previously reported for AHL **1** [32], and the only detectable side product resulted from lactone hydrolysis. Moreover, no epimerization was observed upon similar treatment of AHLs **3a** and **3b**. Thus, AHLs **3a** and **3b** are stable during the assay conditions, and are AHL signals recognized by *A. baumannii*.

### Characterization of AHL 3 Autoinducers in *P. aeruginosa*

We also assessed the activities of AHLs **3a** and **3b** in *Pseudomonas aeruginosa*. Although 3-hydroxy-AHLs have not been isolated from this species, a previous study found that a racemic mixture of AHLs **3** was active as an autoinducer in *P. aeruginosa*; however, this compound was approximately 8-fold less potent than AHL **1** [33]. Moreover, as AHL **1** exhibited partial activity in our *A. baumannii* biochemical assays, we were interested to examine if any crossover activity existed with AHLs **3** [34]. Autoinducer activity assays were conducted using *P. aeruginosa* luminescence reporter strain PAO-JP2, a PAO1 *lasI/rhlI* double mutant (see Supporting Information) [35], [36]. Although AHLs **3a** and **3b** exhibited >200-fold diminished autoinducer activities with respect to AHL **1** (EC_50_ values of 3.13 µM, 2.60 µM and 12.6 nM, respectively), the activities of AHLs **3a** and **3b** were again nearly identical (Figure 5). These results further confirm the insignificance of stereochemistry at the 3-hydroxy position for quorum sensing and possibly implicate some evolutionary stereochemical promiscuity for 3-OH-AHL quorum sensing signaling molecules.

**Figure 5:** Autoinducer activities of AHLs 3a and 3b in comparison to AHL 1 in *P. aeruginosa* strain PAO-JP2. Values shown are relative luminescence units normalized with respect to cell viability (OD_600_). Closed square  =  **1**. Closed circle  =  **3a**. Open circle  =  **3b**.

### Attempt at the Determination of 3-OH Stereochemistry of AHL 3 from *A. baumannii*

In order to determine the natural stereochemistry of the 3-OH substituent of AHL **3** produced by *A. baumannii*, we utilized the recently reported protocol from Schulz and co-workers. Secreted AHL extract was obtained from an overnight culture of *A. baumannii* by extraction with acidified ethyl acetate (0.1% formic acid in ethyl acetate) as previously described [10]. Upon concentration of the crude extract, LC-MS analysis was performed to confirm the presence of AHL **3**. To determine the stereochemistry of the 3-OH position, the homoserine lactone was hydrolyzed to the corresponding methyl ester using acidified methanol for analysis using chiral gas chromatography (GC) as previously reported by Schulz and co-workers. However, even with pure samples of **3a** and **3b**, the reported conditions resulted in racemization of the hydroxyl group. Silylation using BSTFA (N,O-bis(trimethylsilyl) trifluoroacetamide) and TMCS (trimethylchlorosilane) and acetylation of the 3-OH group were also attempted; however, in each case, the resulting product failed to be detected by chiral GC.

## Discussion

To try and elucidate this stereochemical anomaly, we first examined the reported crystal structures of 3-oxo-AHLs bound to quorum sensing-facilitating LuxR-type receptors [37]. While the binding interactions for the lactone and 1-oxo moieties are well conserved and would also likely be conserved in AbaR, deviations have been observed within the chemical sphere of the 3-oxo group [37]. In LasR, the AHL receptor in *P. aeruginosa*, the 3-oxo group of AHL **1** hydrogen bonds with Arg61 via a water molecule [37], [38]. However, in TraR, which recognizes 3-oxo-C_8_-HSL in *Agrobacterium tumefaciens*, the 3-oxo group hydrogen bonds with Thr129 and the main chain of Ala38 [37]. These differences cause the acyl chains to adopt different orientations in the hydrophobic binding tunnels of these receptor proteins. Thus, it is plausible that no conservation exists in the binding of the 3-oxo functionality and therefore, the binding site in AbaR readily accepts either stereoisomer.

The structures of β-hydroxy- and β-ketoamides have also been studied previously using NMR spectroscopy [39], [40]. β-Ketoamides largely exist in the keto tautomeric form unlike their β-ketoester counterparts due to resonance stabilization by the more electron-donating nitrogen heteroatom. This conformation is further stabilized due to reduced steric interactions between the groups flanking the β-ketoamide motif [39], [40]. To minimize possible electrostatic repulsion between the two carbonyl groups, however, the keto tautomer is conformed such that the carbonyls are in an opposed orientation [39]. In fact, a similar orientation was observed in the crystal structure of AHL **1** bound to LasR [38]. Thus, there is little “cross-talk" between the lactone and β-ketoamide portions of AHL **1**. As for β-hydroxyamides, interestingly, by NMR no internal hydrogen bonds have been observed between the hydroxy group and amide carbonyl, both in previous studies [40] and by us (data not shown). This implies that β-hydroxyamides exist in a *trans*-like configuration, and as such, AHLs **3a** and **3b** may be structurally similar to AHL **1** within the receptor's microenvironment with little binding site reorganization required to accommodate either 3-hydroxy stereoisomer.

While *A. baumannii* is classified as a γ-proteobacteria of the order *Pseudomonadales* similar to *P. aeruginosa*, its quorum sensing genes are more closely related to those of environmental strains rather than pathogenic strains and little similarity exists between LasR and AbaR [11]. Phylogenetic studies have indicated that these genes were likely acquired horizontally from *Halothiobacillus neapolitanus*, a sulfur-oxidizing bacterial species of the order *Chromatidales* [11]. Interestingly, however, *A. baumannii* shows no evolutionary relationship with *H. neapolitanus* [11]. As *Acinetobacter* have been shown to readily acquire foreign DNA, including many multidrug resistance genes [41], we would suggest that *A. baumannii* has evolutionarily adopted this unique, yet promiscuous AHL-mediated quorum sensing system to ensure its survival, particularly in the presence of other proteobacteria. This is particularly evident in light of our data demonstrating that AHL **1**, which is not produced by *A. baumannii*, is still ∼50% active as an autoinducer. Although mixed *A. baumannii* biofilms have not been reported such as those identified with *P. aeruginosa* and *Burkholderia cepacia* [34], future research aimed at probing the validity of this hypothesis would be important to determine if *A. baumannii* engages “eavesdropping" to exacerbate its virulence [42]. Additional support for this could stem from the fact that *A. baumannii* was found to produce up to six different AHL signals (Figure 6); however, only one receptor has been identified based on genome mining. It remains to be seen if AbaR is its only quorum sensing receptor and what role other AHL signaling molecules play in this species.

**Figure 6:** AHLs produced by *A. baumannii*.

With respect to our findings, we would like to frame it within the context of other groups working in this area. Firstly, although the observed stereochemical insignificance is unique to AHLs, a similar finding was observed for CAI-1, a non-AHL-based autoinducer produced by *Vibrio cholerae* (Figure 7) [43]. While (*S*)-CAI-1 is the natural autoinducer, both stereoisomers (Figure 7) were generated synthetically and examined in a *V. cholerae* reporter strain [43]. Interestingly, similar to our findings, both the (*R*)- and (*S*)-stereoisomers exhibited very similar autoinducer activities [43]. However, these compounds are not AHLs; thus, our findings are unique for this class of autoinducer. In these regards, for AHLs, a (*R*)-stereocenter at the 3-OH position was observed in all prior stereochemical studies on this class of autoinducer, and the unnatural (*S*)-stereoisomer was found to exhibit little to no activity [15], [16], [20], [21]. Although we were not successful in discerning the stereochemistry of the 3-OH substituent of AHL **3** from *A. baumannii* cell culture, it is likely that it is the (*R*)-stereoisomer in agreement with these previous studies, as 3-OH AHL biosynthesis is believed to be stereoselective [22], [23]. Secondly, we would also like to bring to light the difference between our study and the unnatural AHL analogue syntheses being performed by several laboratories [44]. In our study, we have synthesized a single stereochemical isomer to understand the impact that this position has on quorum sensing in the bacteria from which it is produced, while Blackwell and others [44] are interested in the synthesis of unnatural AHLs through modification of both “head" and “tail" moieties to generate modulators, both agonists and antagonists, of quorum sensing. Thus, we view these studies to be fundamentally different.

**Figure 7:** Structure of (*S*)-CAI-1 produced by *V. cholerae* and its stereoisomer.

In conclusion, we have synthesized both diastereomers of 3-OH-C_12_-HSL, an autoinducer isolated from *A. baumannii*, in order to discern the impact that the 3-position stereochemistry in this AHL has upon quorum sensing. We have discovered that stereochemistry at this position does not appear to play a role in this bacterial signaling process, thus, providing a unique example of stereochemical insignificance for signaling activity. Moreover, as this phenomenon was observed in both *A. baumannii* and *P. aeruginosa*, it is possible that similar findings may be uncovered among other Gram-negative bacteria employing 3-OH-AHLs. The research developed herein is expected to facilitate studies toward developing strategies for combating *A. baumannii* infection including antibodies raised to sequester this quorum sensing signaling molecule [32], [45].

## Methods

### General Materials and Methods

The relative amount of β-galactosidase expressed in each sample was determined using the chemiluminescence-based detection kit Beta-Glo® Assay System (Promega, Madison, WI). All luminescence and absorbance readings were measured on a SpectraMax M2e Microplate Reader (Molecular Devices). All data was analyzed using GraphPad Prism version v5.0b for Mac OS X (GraphPad Software, www.graphpad.com). Data are represented as normalized with respect to the negative control.

### *A. baumannii* β-Galactosidase Assay

A β-Galactosidase assay for *A. baumannii* using a *abaI::lacZ* mutant *A. baumannii* strain, containing an *abaI* promoter fused with a lacZ gene, was employed and adapted to 96-well plate format. Briefly, 200 µL of 1∶1000 diluted overnight culture in modified M9 media (0.2% glucose and 0.5% casimino acids) was added to wells of a 96-well microtiter plate, which were subsequently treated with various concentrations of AHLs at 37°C with shaking until the culture reached mid-log phase. The relative amount of β-galactosidase expressed in each sample was then determined. Following the manufacturer's manual, after equilibrating the cell culture to 25°C for 10 min, 50 µL of cell suspension was transferred from each well to a new opaque 96-well plate and mixed with an equal amount of assay solution. After 1 h incubation at 25°C in the dark, the development of luminescence signal was recorded in relative light units (RLU) and normalized by the original OD_600_ in each well. The ratio of luminescence/OD was plotted against the concentration of compounds to compare the relative activation level of *abaI* promoter. Each concentration of the dose-response curve was analyzed in triplicate simultaneously (i.e. on the same 96-well plate).

## Supporting Information

Scheme S1 Mosher ester synthesis.
(TIF)

Scheme S2 Synthesis of AHL 3 derivative for stability studies.
(TIF)

Figure S1 Conformations used for the analysis of the Mosher esters of 3b.
(TIF)

Figure S2 ^1^H NMR spectral data of 3b-(*S*)-MTPA ester.
(TIF)

Figure S3 ^1^H NMR spectral data of 3b-(*R*)-MTPA ester.
(TIF)

Figure S4 Preparative HPLC spectra of a mixture of 3a and 3b.
(TIF)

Figure S5 ^1^H NMR analysis. •  =  (*S*)-Mosher acid chloride ((*R*)-Mosher acid); □  =  DMAP; ◊  =  Triethylamine; Δ  =  3−[(Diethylamino)propyl]amine.
(TIF)

Figure S6 ^1^H NMR analysis. •  =  (*R*)-Mosher acid chloride ((*S*)-Mosher acid); □  =  DMAP; ◊  =  Triethylamine; Δ  =  3−[(Diethylamino)propyl]amine.
(TIF)

Table S1 Δ*δ* ( = *δ_S_*−*δ_R_*) data for the (*S*)- and (*R*)-MTPA- Mosher esters of 3b.
(TIF)
